This article has been retracted.

# MicroRNA-330 Is an Oncogenic Factor in Glioblastoma Cells by Regulating SH3GL2 Gene

**DOI:** 10.1371/journal.pone.0046010

**Published:** 2012-09-21

**Authors:** Shengtao Qu, Yilong Yao, Chao Shang, Yixue Xue, Jun Ma, Zhen Li, Yunhui Liu

**Affiliations:** 1 Department of Neurosurgery, Shengjing Hospital of China Medical University, Shenyang, People’s Republic of China; 2 Department of Neurobiology, College of Basic Medicine, China Medical University, Shenyang, People’s Republic of China; 3 Institute of Pathology and Pathophysiology, China Medical University, Shenyang, People’s Republic of China; University of Chicago, United States of America

## Abstract

MicroRNAs have recently emerged as key regulators of cancers. This study was therefore conducted to investigate the role of miR-330 in biological behaviors of human glioblastoma U87 and U251 cell lines and its molecular mechanism. SH3GL2 gene was identified as the target of miR-330. MiR-330 overexpression was established by transfecting miR-330 precursor into U87 and U251 cells, and its effects on proliferation, migration, invasion, cell cycle and apoptosis were studied. Overexpression of miR-330 can enhance cellular proliferation, promote migration and invasion, activate cell cycle and also inhibit apoptosis in U87 and U251 cells. Collectively, these above-mentioned results suggest that miRNA-330 plays an oncogenic role in human glioblastoma by regulating SH3GL2 gene and might be a new therapeutic target of human glioblastoma.

## Introduction

With a prevalence of approximately 60%, glioblastoma remains the most common malignant primary brain tumors in adult central nervous system. Despite aggressive surgery, combined radiation and chemotherapy, the median survival time is approximately 14 months [1]. Therefore, how to prolong the survival time of patients of glioblastoma is an urgent problem we are facing. The recent study of miRNAs brings us possibilities for the treatment of human glioblastoma [2], [3].

MicroRNAs (miRNAs) are now recognized as a class of small non-coding RNA molecules throughout the genomes of mammal [4]. They post-transcriptionally regulate protein expression by targeting the 3′-UTR of target mRNA which causes either degradation or repression of translation. Recently many miRNAs are found to play important roles in the development and maintenance of tumorigenesis. A large set of miRNAs are lower expressed or overexpressed in human tumors compared to normal tissues and miRNAs-mediating gene silencing promotes or inhibits tumor cell growth. Such regulators are usually regarded as the enhancers or suppressors of tumor progression. MiR-21 is overexpressed and has been identified as an antiapoptotic factor in human glioblastoma cells [5], [6]. Additionally, miR-128, miR-34a, miR-7 and many other miRNAs also act as tumor suppressors in human glioblastoma cells [7]–[9]. MiR-330 gene was firstly found by Weber in 2005, located at 19q13.32 [10] **.** Previous studies show that miR-330 was able to acts as tumor suppressor and induced apoptosis of prostate cancer cells through E2F1-mediated suppression of Akt phosphorylation [11]. However, the function and molecular mechanism of miR-330 in determining the malignant phenotype of human glioblastoma are less elusive.

SH3GL2 gene is a candidate tumor suppressor gene that particularly more highly expressed in central nervous system [12], [13]. Moreover, decreased expression of SH3GL2 is shown to be associated with tumorigenesis of laryngeal carcinoma [14]. Our previous study has shown that SH3GL2 gene is obviously less expressed in human glioblastoma which indicates the correlation of its expression with the incidence of glioblastoma [15]. Potter, et al also observed deletion of the locus in pilocytic astrocytomas suggesting a tumor suppressor role of SH3GL2 in brain tumors [16]. However, the underlying mechanism is still unclear. The recent prediction of miR-330 targeting SH3GL2 3′-UTR has led our further study on the mechanism of downregulation of SH3GL2 gene in glioblastoma.

Here, for the first time, we uncovered a comprehensive analysis of the regulation of miR-330 and SH3GL2 expression in glioblastoma. We investigated the regulatory effects of miR-330 on SH3GL2 and explored the potential oncogenic mechanism of miR-330 in glioblastoma cells.

## Materials and Methods

### Human Tissue Samples

All human normal brain and glioma tissue samples were obtained from the Department of Neurosurgery, Shengjing Hospital of China Medical University. This study procedure was approved by The Institutional Review Board at the hospital. All participants provided written informed consent. The tissue samples were obtained from those without necrosis and coagulation parts. For each sample, the major portion of tissue was frozen immediately in liquid nitrogen for molecular analysis, and the remaining tissue was fixed in paraformaldehyde for histological examination. All samples were histologically classified and graded according to WHO guidelines by tow experienced clinical pathologists.

### Reagents and Cell Culture

Dulbecco's Modified Eagle Medium: Nutrient Mixture F-12 (DMEM/F12) and fetal bovine serum (FBS) was purchased from Gibco (Carlsbad, CA, USA). Trizol and Lipofectamine™ 2000 transfection reagent were purchased from Invitrogen (Carlsbad, CA, USA). MicroRNAs and their negative control molecules were synthesized by Ambion (Austin, TX, USA). The siRNA targeting SH3GL2 gene and its negative control molecules were synthesized in vitro using the Ambion Silencer ™ siRNA Construction Kit. All other chemicals and reagents were purchased from Sigma-Aldrich (Shanghai, China) unless otherwise specified. Human glioblastoma cell lines U87 and U251 were obtained from the Chinese Academy of Medical Sciences and cultured in DMEM/F12 medium supplemented with 10% fetal bovine serum (FBS), 100 units of penicillin/ml and 100 ng of streptomycin/ml. HEK-293 cells were also from the Chinese Academy of Medical Sciences and cultured in DMEM medium of high glucose without penicillin and streptomycin. All cells were incubated in a 5% CO_2_ humidified incubator at 37°C.

### Vector Construction

The 3′-UTR sequence of human SH3GL2 gene was amplified by PCR using the following primers: SH3GL2 forward primer, 5′-TCG AGG ATG TTA TGC TGG CTG-3′; SH3GL2 reverse primer, 5′-CTG CGG CCT GCA CTT GGG ATGT-3′. For its mutagenesis, the sequence complementary to the binding site of miR-330 in its 3′-UTR (TGC TTT G) was replaced by GAA GCC A using the overlap PCR method. The wild type and mutant type 3′-UTRs of SH3GL2 were cloned into pmirGLO Dual-Luciferase miRNA target expression vector using the Xho I and Sal I sites. These constructs were validated by sequencing.

### Cell Transfection

Cells at 50–70% confluence were transfected using lipofectamine 2000 reagent (Invitrogen, CA, USA) 24 h after plating. Transfection complexes were prepared according to the manufacturer’s instructions and added directly to the cells to a final oligonucleotide concentration of 50 nmol/L. At 6 h after the transfection, the medium was replaced with fresh DMEM/F12 with 10% fetal bovine serum, and the cells were incubated for an additional 48 h or 72 h. Then the transfected cells were harvested for further study. Those transfected with miRNA precursors were divided into 5 groups: mock group with no miRNA precursor but PBS, pre-miR-con group with pre-miR negative control precursor, pre-miR-330 group with miR-330 precursor, anti-miR-con with anti-miR negative control precursor and anti-miR-330 group with miR-330 inhibitor precursor. Those transfected with siRNA were divided into 2 groups: siRNA control (siRNA-con) group and siRNA-SH3GL2 group.

### Bioinformatics Method and Luciferase Reporter Assay

The common targets of miR-330 predicted by computer-aided algorithms were obtained from multiple target prediction programs: Targetscan and Miranda (http://www.targetscan.org/and http://www.microrna.org/). HEK-293 cells were seeded into a 24-well plate. After cultured overnight, cells were co-transfected with the wild-type or mutated SH3GL2 3′-UTR reporter plasmid, and transfected with pre-miR-330 or pre-miR-con precursors. Luciferase assays were performed 48 h after transfection using the Dual-Luciferase Reporter Assay System (Promega, WI, USA).

### RNA Extraction, Reverse Transcription PCR and Quantitative Real-time PCR

Total RNA of each group was extracted from the cells using Trizol according to the manufacturer’s instruction. RT-PCR was conducted using an RT-PCR kit (TaKaRa, Dalian, China). The primers used were all synthesized by Sangon (Shanghai, China). To analyze miR-330 expression levels, the stem-loop RT-PCR assay was used to quantify the miRNAs expression levels. The RT-PCR primers were as following: miR-330 RT primer: 5′-GTC GTA TCC AGT GCG TGT CGT GGA GTC GGC AAT TGC ACT GGA TAC GAC TCT CTG C-3′. MiR-330 PCR primers are: forward: 5′-CGG CAA AGC ACA CGG CCT G-3′; reverse: 5′-TGC GTG TCG TGG AGT CGG C-3′. U6 RT primer is: 5′-TGG TGT CGT GGA GTC G-3′. U6 PCR primers are: forward: 5′-CTC GCT TCG GCA GCA CA-3′; reverse: 5′-AAC GCT TCA CGA ATT TGC GT-3′. qRT-PCR was performed using SYBR Premix Dimer Eraser (TaKaRa, Dalian, China) on a 7500HT system. The expression levels of miR-330 were normalized with reference to expression levels of U6, and fold changes were calculated by relative quantification (2^−ΔΔCt^). The primer sequences for SH3GL2 gene expression were as follows: β-actin forward: 5′-ATC ATG TTT GAG ACC TTC AAC A-3′, reverse: 5′-CAT CTC TTG CTC GAA GTC CA-3′; SH3GL2, forward: 5′-GGC CCT GTC ACT CCT GAG AT-3′, reverse: 5′-GGC ATC CAG GTT ATC GGG GA-3′; Amplification was performed over 35 cycles: 94°C/60 s (denaturation), 58°C/45 s (annealing) and 72°C/45 s (extension). The relative SH3GL2 mRNA levels were normalized to those of β-actin mRNA levels using Quality One analysis software (Bio-Rad, USA).

### Western Blot Analysis

Total protein from transfected cells was extracted in RIPA buffer supplemented with protease inhibitors (100 mM Tris, pH 7.4, 150 mM NaCl, 5 mMEDTA, 1% Triton X-100, 1% deoxycholate acid, 0.1% SDS, 2 mM phenylmethylsulfonyl fluoride, 1 mM sodium orthovanadate, 2 mM DTT, 2 mM leupeptin, 2 mM pepstatin). The samples were centrifuged (12,000 g, 4°C) for 20 min and the protein concentration was determined by the BCA method (Beyotime Institute of Biotechnology, Jiangsu, China). The proteins were separated using 12% SDS-PAGE and then electrophoretically transferred to a PVDF membrane (Millipore, USA). The membranes were blocked in blocking buffer (5% non-fat milk dissolved in Tris-buffered saline-Tween, TBS-T) overnight at 4°C. The blots were then incubated with mouse monoclonal anti-SH3GL2 antibody (diluted 1∶500, Santa Cruz Biotechnology, CA, USA) and mouse monoclonal anti-β-actin antibody (diluted 1∶4000, Santa Cruz Biotechnology). Protein bands were visualized by ECL (Santa Cruz Biotechnology, CA, USA) and detected by ECL Detection Systems (Thermo Scientific). The relative integrated density values (IDVs) were calculated based on β-actin protein as an internal control.

### Proliferation Assay

U87 and U251 cells were seeded into 96-well plates at a density of 2000 cells/well with five replicate wells for each group, transfected and assayed 24, 48, 72, 96, 120 h after transfection. 20 µl of MTT (5 mg/ml) was added into each well and incubated for another 4 h, and then the supernatant was discarded, 150 µl of DMSO was added to each well to dissolve the precipitate. Optical density (OD) value was measured at the wavelength of 490 nm every 24 h for 5 consecutive days after treatment. The data were derived from three independent experiments.

### Cell Migration and Invasion Assay

Migration of U87 and U251 cells was assayed using chamber (Costar, USA) with polycarbonic membrane (6.5 mm in diameter, 8 µm pore size). Cells were grown to about 70% confluence and transfected with the desired miRNAs. After 24 h, the cells were replaced with serum-free medium incubated for another 24 h. Then cells were trypsinized and collected. 5×10^4^ cells in serum-free medium were added to the upper chamber. Then 600 µl medium with 10% FBS was added to the lower chamber. Cells were incubated for 24 h at 37°C, and then non-migrating cells on the top of membrane were removed with cotton swabs. Cells that migrated to the bottom of the membrane were then fixed with methanol and stained with 20% Giemsa solution for 30 min at 37°C and washed twice with PBS. Then stained cells were subjected to a microscopic inspection counted within five randomly chosen fields and the average number was taken. For the cell invasion ability assay, the procedure was similar to migration assay, but the transwell membrane was coated with a 500 ng/µl Matrigel solution (BD, Franklin Lakes, NJ), and incubated for 4h at 37°C then collected the after-transfected cells added to the upper chamber for the further assay. Invasive cells were fixed, stained with 5% crystal violet and counted as previously described.

### Cell Cycle Assay

To assess the effect of miR-330 on the cell cycle, the U87 and U251 cells were transfected with pre-miR-con and pre-miR-330. Briefly, 72 h after transfection 1×10^6^ cells were washed with phosphate buffer saline (PBS), trypsinized and resuspended in ice-cold PBS. Cells were then gently pelleted by centrifugation (500 g for 5 min at 4°C), the supernatant was removed and the cells were fixed and permeabilized in 70% ethanol at −20°C. Fixed cells were washed with PBS and incubated in the dark for 30 min with a propidium iodide (PI) staining solution containing 50 µg/ml propidium iodide (PI) and 100 µg/ml RNase A in PBS. The cells were then analyzed for DNA content on a FACscan (BD FACSCalibur, USA) and G0/G1, S and G2/M fractions were determined.

### Apoptosis Assay

The effect of miR-330 expression on cell apoptosis was assessed by Annexin V-FITC/PI staining. U87 and U251 cells were transfected with mock, pre-miR-330, anti-miR-330 and their negative control molecules for 72 h. Then, the cells were harvested and stained with Annexin V-FITC and PI according to the instruction of the manufacturer. Cell samples were analyzed on a FACsan and apoptotic fractions were determined.

### Statistical Analysis

For all the experiments, data were obtained from three independent experiments. All results were expressed as the mean ± SD for each group. Data were analyzed by use of SPSS 13.0 software. When appropriate, two group comparisons were analyzed with a *t*-test and more than two groups comparisons were analyzed with one-way ANOVA. P<0.05 was considered significant and symbolized by an asterisk in the graphs.

## Results

### MiR-330 Expression was Increased in Glioblastoma

To determine the levels of miR-330 in established glioblastoma cell lines, glioblastoma tissues and normal brain tissues, total RNAs were extracted from U87, U251 and U373 cells, glioblastoma tissues and normal brain tissues. The expression levels of miR-330 were analyzed using RT-PCR and quantitative real-time PCR**.** U6 RNA level was used as an internal control. As shown in Figure 1, the expression levels of miR-330 normalized to U6 were significantly up-regulated in five glioblastoma tissues and three glioblastoma cells when compared to the three normal brain tissues. This result indicates that miR-330 is up-regulated in glioblastoma.

**Figure 1:** MiR-330 was overexpressed in human glioblastoma tissues and cells. Relative miR-330 expression levels were analyzed by qRT-PCR in normal brain tissues, glioblastoma tissues and established glioblastoma cell lines. U6 RNA level was used as an internal control. Asterisks indicate significant difference when compared to normal brain tissues (P<0.05).

### MiR-330 Directly Targeted the 3′-UTR of SH3GL2

Bioinformatics analyses available on the public miRNA databases were used (http://www.targetscan.org/and http://www.microrna.org/) to identify miRNAs that specifically target SH3GL2. MiR-330 was shown to have a putative binding site to the 3′-UTR region of SH3GL2 with 100% conserved sequence. A highly conservative miR-330 binding site at SH3GL2 3′-UTR 56–62 base position was predicted in many species, such as the *H. Sapiens*, the *M. muculus* and the *R. Norvegius et al*. The seed for miR-330 to SH3GL2 3′-UTR is shown in Figure 2A. The wild type of SH3GL2 3′-UTRs was cloned into pmirGLO Dual-Luciferase miRNA target expression vector. Overexpression of miR-330 decreased luciferase activity of this reporter to about 60% of the control level (Figure 2C), suggesting that miR-330 inhibits the 3′-UTR function of SH3GL2. To test whether miR-330 specifically inhibited SH3GL2 by its potential binding site of seed sequence, the mutated reporter at miR-330 binding site was constructed (Figure 2B). Forced expression of miR-330 did not affect the mutant SH3GL2 reporter activities (Figure 2D). These results indicate that SH3GL2 is a direct target of miR-330 with the specific binding site at the seed sequence.

**Figure 2:** MiR-330 negatively regulated SH3GL2 through binding to the 3′-UTR of SH3GL2. (A) Schematic diagram of putative miR-330 binding site in the 3′-UTR of SH3GL2 in human. The seed sequence of miR-330 matches 3′-UTR of SH3GL2 (in bold). (B) The corresponding mutated nucleotides of the SH3GL2 3′-UTR was labeled in bold bellow. (C) Relative luciferase activities of SH3GL2 wild type 3′- UTR were obtained by co-transfection of PBS (mock), negative control miRNA or miR-330 precursors; and calculated as the ratio of firefly/renilla activities in the cells and normalized to those of the control. The results were presented as mean±SD from three independent experiments with each experiment in triplicate. Asterisk indicates significant difference when compared to control (P<0.05). (D) Relative luciferase activities of pmirGLO plasmid, SH3GL2 wild type and mutant type 3′- UTR were obtained by co-transfection of miR-330 precursor; and calculated as the ratio of firefly/renilla activities in the cells and normalized to those of the control. The results were presented as mean±SD from three independent experiments with each experiment in triplicate. Asterisk indicates significant difference when compared to control (P<0.05).

### MiR-330 Post-transcriptionally Inhibited SH3GL2 Expression

The relationship between miR-330 level and SH3GL2 expression was analyzed in U87 and U251 cells. When cell lines were transfected with exogenous miR-330 and its inhibitors, the level of SH3GL2 protein was detected by western blotting. As shown in Figure 3B **,** there was a significant inverse correlation between miR-330 and SH3GL2 protein level in the pre-miR-330 group versus pre-miR-con group (P<0.05), while there was no obvious difference between mock group and pre-miR-con group. What’s more, the anti-miR-330 played the opposite effect of pre-miR-330 with an increasing level of SH3GL2 protein expression versus either pre-miR-330 or anti-miR-con group (P<0.05). Meanwhile, the SH3GL2 mRNA level after transfection in each group was also detected by RT-PCR. However, there was no statistical significance among the five groups (Figure 3A). As shown in Figure 3, miR-330 induced a significant decrease of SH3GL2 protein expression without influence on mRNA level. To further validate the effect of miR-330 on SH3GL2 gene, rescue experiment by siRNA on SH3GL2 in U87 cells was performed. As shown in Figure S1, there were decreases at both mRNA and protein level of SH3GL2 gene (P<0.05). All of these results indicate that miR-330 post-transcriptionally inhibits SH3GL2 expression and miR-330 is negatively correlated with SH3GL2 protein expression in glioblastoma cells.

**Figure 3:** MiR-330 regulated SH3GL2 expression at the post-transcriptional level. (A) Overexpression of miR-330 or transfection of exogenous miR-330 inhibitor did not change the SH3GL2 mRNA level detected by RT-PCR. The effectiveness of miR-330 on SH3GL2 mRNA was analyzed by RT-PCR. The mRNA levels of the SH3GL2 were shown and normalized against that of β-actin. (B) Overexpression of miR-330 inhibited SH3GL2 expression at protein level. The expression level of SH3GL2 and β-actin in U87 and U251 cells transfected with exogenous miR-330 or its inhibitor were analyzed by Western blot 48 h after transfection. β-actin was used as an internal loading control (P<0.05). Accompanying graphs show densitometry analysis of SH3GL2 expression. Data are means of three independent experiments ± SD.* P<0.05 compared with control group.

### MiR-330 Promoted Cellular Proliferation of Glioblastoma

To investigate whether miR-330 could influence glioblastoma cell proliferation, MTT assay was performed in U87 and U251 cells. The result demonstrated that U87 and U251 cells transfected with pre-miR-330 exhibited a significant increase of cellular viability compared with cells treated by pre-miR-con (P<0.05). While, there was no significant difference between mock group and pre-miR-con group in both cell lines. On the contrary, anti-miR-330 decreased cellular proliferation in both U87 and U251 cells compared with anti-miR-con group (Figure 4). In the rescue experiment, U87 cells transfected with siRNA-SH3GL2 showed higher cellular proliferation than that of siRNA-con group (Figure S2A). These results demonstrate that miR-330 can promote cellular proliferation in glioblastoma cells in an SH3GL2-dependent way.

**Figure 4:** MiR-330 increased cell proliferation of U87 and U251 cells. MTT assay showed that U87 (A) and U251 (B) cells transfected with pre-miR-330 proliferated at a higher rate than the pre-miR-con group (P<0.05). Those transefected with anti-miR-330 group showed a lower proliferation rate than the anti-miR-con group (P<0.05).There was no obvious difference between mock group and the two control groups in the experiment. Values represent the mean ± SD of three independent experiments.* P<0.05 compared with control group.

### MiR-330 Increased Glioblastoma Cell Migration and Invasion

To examine whether overexpression of miR-330 affected the migration and invasion capacity of glioblastoma cells, transwell assays were introduced. We observed that miR-330 overexpression enhanced FBS-induced migration ability of glioblastoma cells compared with pre-miR-con group (P<0.05) (Figures 5A and 5C). In parallel, a Matrigel invasion assay was also performed to study the effects of miR-330 on the invasion of glioblastoma cells. The results clearly revealed that miR-330 also increased FBS-induced invasion of U87 and U251 cells compared with pre-miR-con group (P<0.05) (Figures 5B and 5D). However, there was no significant difference between mock group and pre-miR-con group. We also found the opposite effects of anti-miR-330 exerted on both cell lines compared with anti-miR-con or pre-miR-330 group (P<0.05). While the U87 cell showed higher migration and invasion capacity in siRNA-SH3GL2 group than in siRNA-con group (P<0.05) (Figure S2B).These results above strongly suggest that miR-330 is an important factor involved in the migration and invasion of glioblastoma cells by regulating SH3GL2 gene.

**Figure 5:** MiR-330 increased migration and invasion of U87 and U251 cells. U87 and U251 cells were transfected miRNA precursors and then subject to transwell migration and invasion assays. After 24 h and 48 h, migration and invasion cells were correspondingly counted after staining with Giemsa (A and B) or 5% crystal violet (C and D). Representative photographs of migration and invasion cells on the membrane and accompanying statistical plots were presented. There were obvious differences between pre-miR-330 group and pre-miR-con group; the anti-miR-330 group showed a contrary effect compared with mock, negative control and pre-miR-330 groups (P<0.05). However, there was no obvious difference between mock group and negative control groups. Values represent the mean ± SD from three independent experiments.* P<0.05 compared with control group.

### MiR-330 Accelerated Glioblastoma Cell Cycle

The cell cycle distribution of the cells treated with miR-330 was examined using flow cytometry. The results showed that there were higher S, G2/M phase fractions in glioblastoma cells transfected with pre-miR-330 compared with the cells transfected with pre-miR-con (P<0.05) (Figure 6). In the rescue experiment, the cell cycle distribution between siRNA-SH3GL2 group and siRNA-con group showed a significant difference (P<0.05) (Figure S3A). These data suggest that overexpression of miR-330 cause acceleration of cell cycle through influencing SH3GL2 gene.

**Figure 6:** MiR-330 promoted cell cycle progression of U87 and U251 cells. Cell cycle distribution of U87 and U251 cells transfected with pre-miR-con and pre-miR-330. The percentage of cells in the different cell cycle phases was plotted, and the results represent the mean ± SD. * P<0.05 compared with control group.

### MiR-330 Inhibited the Apoptosis of Glioblastoma

To confirm that the overexpression of miR-330 was associated with apoptosis, we examined the apoptosis of the cells by flow cytometry 72 h after transfection. The results obviously demonstrated that there was a significant decrease of apoptosis in glioblastoma cells transfected with pre-miR-330 compared with cells transfected with pre-miR-con (P<0.05). While those transfected with anti-miR-330 showed an increase of apoptosis compared with anti-miR-con and pre-miR-330 groups (P<0.05) (Figure 7). In the rescue experiment, the siRNA-SH3GL2 group also showed a lower apoptotic proportion than the siRNA-con group (P<0.05) (Figure S3B). These data confirm that miR-330 plays an antiapoptotic role in glioblastoma cells by regulating SH3GL2 gene.

**Figure 7:** MiR-330 inhibited apoptosis of U87 and U251 cells. Apoptosis of U87 and U251 cells were monitored by flow cytometry. Early apoptotic cells are Annexin V+/PI−, late apoptotic cells are Annexin V+/PI+, necrotic cells are Annexin V−/PI+ and healthy cells are Annexin V−/PI−. A representative experiment of three performed was shown. The percentage of apoptotic cells is indicated and the results represent the mean ± SD. * P<0.05 compared with control group.

## Discussion

In this study, we firstly revealed the oncogenic role of miR-330 in human glioblastoma cells and its relationship with SH3GL2 gene. We found that miR-330 could influence the proliferation, migration, invasion, cell cycle and apoptosis of human glioblastoma by regulating SH3GL2 gene.

SH3GL2, also termed as endophilin-1, is a multifunctional gene [17]. SH3GL2 mainly distributes in central nervous system, particularly enriched in the presynaptic ganglion [12]. Besides its endocytic functions, the non-endocytic functions of SH3GL2 may play a more important part in the malignant progression of tumor. Previous studies have shown that SH3GL2 gene is expressed less and functions as a tumor suppressor gene in many different tumor tissues. Gene chip demonstrated that the SH3GL2 gene expression was significantly decreased in laryngeal cancer. Clinical evidences also showed that there is a reduction of SH3GL2 expression in the samples from the follow-up patients [14]. Osterberg also proved that low expression of SH3GL2 was associated with increased chemotherapy resistance in ovarian cancer [18]. Sinha confirmed the decreased SH3GL2 gene expression in breast cancer [19]. In addition, it was reported that the SH3GL2 gene was involved in head and neck dysplastic lesions [20]. Our previous study found that the SH3GL2 expression was obviously lower in glioblastoma tissues compared with normal brain tissues [15]. These suggest that the SH3GL2 gene may also be a tumor suppressor gene and plays an important role in human glioblastoma. However, the underlying mechanism is still unclear.

Recently, miRNAs have been rapidly developed as potential important molecular markers for cancer and other diseases [21]–[23]. They are found to regulate apoptosis, proliferation, differentiation, development, and metabolism in worm, fly, fish, mouse and human cells [24]. Many studies have shown that miRNAs function as oncogenes or tumor suppressor genes [25]–[27]. MiR-34a is repressed and promotes tumorigenesis in proneural malignant gliomas [28]. Inhibition of the highly expressed miR-221 and miR-222 impairs the growth of prostate carcinoma xenografts in mice [29].

To explore whether there were some microRNAs involved in the regulation of SH3GL2, we applied bioinformatics method (TargetScan and Miranda) to search for the possible microRNAs that target SH3GL2**.** We found that there was a binding site of miR-330 in the 3′-UTR of SH3GL2, suggesting SH3GL2 as a potential target of miR-330. Subsequently, luciferase reporter assay confirmed the prediction of miR-330′s targeting on the 3′-UTR of SH3GL2 gene. Meanwhile, we found a higher relative expression level in glioblastoma tissues and established glioblastoma cell lines than that of normal brain tissues. By transfection of exogenous miR-330, we detected a reduction of SH3GL2 protein expression in two glioblastoma cells. Glioblastoma cells transfected with anti-miR-330 showed higher expression of SH3GL2 protein level. Neither of these miRNA precursor transfections affected the SH3GL2 mRNA level. Meanwhile, we revealed that overexpression of miR-330 could increase the viability of glioblastoma cells. We also found that miR-330 obviously increased migration and invasion of glioblastoma cells. Besides, miR-330 could also influence the cell cycle and act as an antiapoptotic factor in both cell lines. What’ more, we found the opposite effects by transfecting anti-miR-330 precursor. To further confirm the biological behavior change of glioblastoma cells through miR-330′s regulation of SH3GL2, we also transfected the siRNA targeting on SH3GL2 and got similar results as miR-330. In line with the previous studies, these results indicated that miR-330 functioned as an oncogenic miRNA by negatively regulating the candidate tumor suppressor gene SH3GL2 in human glioblastoma cells.

Since the close relationship between miR-330 and the SH3GL2 gene, we analyzed the potential mechanism of this process according to the previous studies. SH3GL2 can regulate intracellular transit and maturation of metalloprotease disintegrin by binding to its cytoplasmic tail, and then affects cell adhesion and growth factor signaling [30]. When binding to Cbl-interacting protein of 85 kDa (CIN85) and Cbl, SH3GL2 can also influence internalization, degradation and intracellular signaling of tyrosine kinase receptors for hepatocyte and epidermal growth factors [31]–[33]. At the same time, this complex mediates ligand-induced downregulation of c-Met and EGF receptors [31], [34]. Both c-Met and EGF receptors cause the development of cancers by influencing their differentiation, proliferation, migration, invasion, cell cycle progression and apoptosis, etc. Hence, SH3GL2 may play a key role in the progression of malignant tumors as a tumor suppressor gene.

A recent study showed that miR-330 induced apoptosis in prostate cancer cells through E2F1-mediated suppression of Akt phosphorylation [11]. Our study showed that exogenous overexpression of miR-330 caused some opposite biological behavior changes in glioblastoma cells compared with those in prostate cancer cells. However, it has been reported that even the same miRNA targets the same gene, which may show different biological effects in different tissues [35]. Hodzic reported that miR-330 post-transcriptionally regulated the expression of deoxycytidine kinase by targeting its 3′-UTR and decreased its sensitivity to gemcitabine in cancer cells [36]. Though, by targeting different gene and maybe through different pathways, miR-330 seems to exert the same effect in this report and our study to some extent. What is to be explored next is the molecular mechanism, downstream signal pathway of SH3GL2 mediates apoptosis and whether there is some crosstalk between other genes and signal pathways. Moreover, in vivo studies are to be performed to validate these findings.

In conclusion, this is the first study to show that the tumor suppressor gene SH3GL2 is negatively regulated by miR-330 at the posttranscriptional level. We also showed that overexpression of miR-330 played an oncogenic role by inhibiting SH3GL2 and affected cell proliferation, migration, invasion and activation of cell cycle in U87 and U251 cells. MiR-330 is a potential novel oncogenic miRNA in glioblastoma and provides a new therapeutic target of human glioblastoma.

## Supporting Information

Figure S1 **Inhibition of SH3GL2 expression by siRNA in U87 cells.** U87 cells were transfected with SH3GL2 siRNA (siRNA-SH3GL2) and its scramble control (siRNA-con) oligonucleotides. Both mRNA and protein levels lower expression of SH3GL2 were revealed compared with scramble control group. * P<0.05 compared with control group.
(TIF)

Figure S2 **Effect of SH3GL2 knocked-down on U87 cell proliferation, migration and invasion.** (A) The proliferation of siRNA-con and siRNA-SH3GL2 transfected U87 cells was analyzed by MTT assay. The cell proliferation rate of siRNA-SH3GL2 group was much higher than that of siRNA-con group. (B) Transwell assay was performed to evaluate the migration and invasion capacity in U87 cells. The migration and invasion capacity of siRNA-SH3GL2 cells was larger than that of siRNA-con group. * P<0.05 compared with control group.
(TIF)

Figure S3 **Effect of SH3GL2 knocked-down on U87 cell cycle and apoptosis.** The cell cycle distribution of siRNA-con and siRNA-SH3GL2 transfected cells was analyzed by flow cytometry. The percentage of cells in the different cell cycle phases was plotted, and the results represent the mean ± SD. * P<0.05 compared with control group. (B) Apoptosis of U87 cells were monitored by flow cytometry after transfected with siRNA to SH3GL2. Early apoptotic cells are Annexin V+/PI−, late apoptotic cells are Annexin V+/PI+, necrotic cells are Annexin V−/PI+ and healthy cells are Annexin V−/PI−. A representative experiment of three performed was shown. The percentage of apoptotic cells is indicated and the results represent the mean ± SD. * P<0.05 compared with control group.
(TIF)
